RETRACTED

# The lncRNA SNHG5‐mediated miR‐205‐5p downregulation contributes to the progression of clear cell renal cell carcinoma by targeting ZEB1

**DOI:** 10.1002/cam4.3052

**Published:** 2020-04-12

**Authors:** Wei Xiang, Lei Lv, Gaofeng Zhou, Wei Wu, Jingdong Yuan, Chuanhua Zhang, Guosong Jiang

**Affiliations:** ^1^ Department of Urology Wuhan No. 1 Hospital Tongji Medical College Huazhong University of Science and Technology Wuhan China; ^2^ Department of Urology Union Hospital Tongji Medical College Huazhong University of Science and Technology Wuhan China

**Keywords:** ccRCC,non‐coding RNAs, ceRNA,ZEB1,miR‐205‐5p, SNHG5

## Abstract

Recent findings have unraveled the critical functions of the long noncoding RNA (lncRNA) SNHG5 in human malignancies. Nevertheless, the role and mechanism of SNHG5 in clear cell renal cell carcinoma (ccRCC) are still elusive. In our study, substantially higher abundance of SNHG5 was observed in ccRCC specimens and cell lines, and increased SNHG5 expression was intimately correlated with tumor size, tumor‐node‐metastasis (TNM) stage, lymph node invasion, and distant metastases in patients with ccRCC. SNHG5 knockdown obviously suppressed the proliferative, migratory, and invasive capabilities of ccRCC cells, whereas SNHG5 overexpression induced the opposite effects. Mechanistically, SNHG5 activated the transcription of ZEB1, which exerts a pivotal role in modulation of epithelia‐mesenchymal transition (EMT) and tumor metastasis. SNHG5 was then shown to act as an endogenous sponge for miR‐205‐5p, which targets ZEB1 in ccRCC. Moreover rescue experiments revealed that SNHG5 promotes ccRCC cell proliferation, migration, and invasion in a miR‐205‐5p‐dependent manner. Additionally, in vivo assays further indicated that overexpression or silencing of SNHG5 in ccRCC cells promoted or suppressed the tumorigenesis and metastasis, respectively*.* Altogether, the present data provide the first evidence that the lncRNA SNHG5 has an oncogenic role in ccRCC through the SNHG5/miR‐205‐5p/ZEB1 signaling axis and represents a novel potential therapeutic regimen against ccRCC.

## Graphical abstract

SNHG5 was found to be highly expressed in ccRCC tissues and cell lines and was intimately associated with TNM stage, lymphatic invasion, and metastasis in patients with ccRCC. Overexpression of SNHG5 facilitates ccRCC progression, whereas knockdown of SNHG5 exerts the opposite effect. SNHG5 acts as a ceRNA to sponge miR‐205‐5p and alleviates the inhibition of miR‐205‐5p on its target ZEB1 in ccRCC.

## 1 INTRODUCTION

Renal cell carcinoma (RCC) is a common form of urological tumors, accounting for nearly 3% of human malignancies worldwide.^1^ Based on histological and cytogenetic features, clear cell renal cell carcinoma (ccRCC) has been demonstrated to be the most common subtype of RCC.^2^ Due to resistance to traditional chemo‐ and radiotherapeutic strategies, surgical removal is still the primary treatment option for ccRCC. However, ccRCC patients exhibit a poor prognosis owing to the high incidence of recurrence and metastasis. Approximately 25% of ccRCC patients will experience local relapse or distant metastasis after surgical operation.^3^, ^4^ Thus, further exploration of the underlying mechanisms of ccRCC development will help to develop more effective target therapies for advanced ccRCC and is of great significance.

RETRACTED

It has been well documented that the dysregulation of long noncoding RNAs (lncRNAs) can contribute to the tumorigenesis and development of human carcinomas. LncRNAs are defined as a subgroup of noncoding RNAs with lengths larger than 200 bp. LncRNAs play vital roles in the processes of transcriptional regulation, posttranscriptional modulation, and epigenetic modification and thus affect biological behaviors of human cancer cells. For example, increased lncARSR expression was found in primary renal tumor‐initiating cells and correlated with poor prognosis in ccRCC patients.^5^ PVT1 was identified as an oncogene that could promote metastasis and predict unfavorable prognosis in patients with ccRCC.^6^ The aberrant expression of HOTAIR was also confirmed to promote ccRCC malignancy by several groups.^7^, ^8^, ^9^, ^10^ Additionally, the overexpression of MALAT1 has been demonstrated to have an oncogenic function in ccRCC via EZH2 and the interaction of MALAT1 with miR‐205.^11^ In contrast, lncRNA‐SARCC has been found to suppress the progression of ccRCC by altering the androgen receptor (AR)/miR‐143‐3p signaling axis.^12^ Notably, a newly reported lncRNA, small nucleolar RNA host gene 5 (SNHG5), was confirmed to exert a critical influence on the occurrence and development of several kinds of human carcinomas, including hepatocellular carcinoma, bladder carcinoma, colorectal cancer, and chronic myeloid leukemia.^13^, ^14^, ^15^, ^16^ However, to the best of our knowledge, whether SNHG5 has a vital influence on the function of ccRCC cells remains elusive.

In this study, we checked the expression of SNHG5 in ccRCC specimens and cell lines and placed a special emphasis on the mechanism of SNHG5 in ccRCC. Elevated expression of SNHG5 was shown in both ccRCC tissues and cell lines. Deregulation of SNHG5 was demonstrated to affect the miR‐205‐5p/ZEB1 signaling axis, which has been implicated in modulating the proliferation, migration, and invasion of ccRCC cells. Based on these findings, the current investigation may reveal novel biomarkers or targeted therapies for ccRCC.

RETRACTED

## 2 MATERIALS AND METHODS

### 2.1 Hierarchical cluster analysis and specimen collection

LncRNA expression data were acquired from The Cancer Genome Atlas (TCGA) database. SNHG5 expression levels between ccRCC (n = 542) and para‐cancerous tissues (n = 68) were compared using hierarchical cluster analysis. Fifty‐two ccRCC tissues and matched nontumor kidney tissues were acquired from individuals who underwent radical nephrectomy and were ultimately diagnosed with ccRCC based on histopathological evaluation at Wuhan No. 1 Hospital, Huazhong University of Science and Technology, between January 2013 and October 2016. All patients were previously untreated, and informed patient consent was recorded in writing. The study was performed complying with the ethical standards of the Helsinki Declaration and ethical approval was received from the ethics committee of Wuhan No. 1 Hospital. Detailed information was exhibited in Table 1. The tissue samples were collected during surgery and snap‐frozen using liquid nitrogen, then stored at −80°C.

**Table 1:** Relationship between SNHG5 expression and clinicopathologic parameters of ccRCC patients

Expression of SNHG5 in ccRCC				
Characteristics	Number of cases	Low	High	*P*‐value
Overall	52	n = 14	n = 38	
Sex				
Male	38	10	28	.8708
Female	14	4	10	
Age(y)				
≤60	15	6	9	.1759
>60	37	8	29	
Tumor size (cm)				
≤4	17	10	7	**.0003** **
>4	35	4	31	
Fuhrman grade				
G1‐G2	37	12	25	.1595
G3‐G4	15	2	13	
TNM stage				
I	26	11	15	**.0124** *
II‐IV	26	3	23	
Lymphatic invasion				
Negative	32	12	20	**.0296** *
Positive	20	2	18	
Distant metastasis				
Absent	37	13	24	**.0360** *
Present	15	1	14	

Abbreviations: M, describes distant metastasis; N, describes adjacent lymph nodes that are involved; TNM, T describes the size of original tumor and whether it has invaded nearby tissue.

Bold value indicates a significant difference.

* *P* < .05,

** *P* < .01

### 2.2 Cell culture

Human RCC cell lines ACHN and 786‐O were acquired from the American Type Culture Collection (ATCC) and maintained in RPMI‐1640 medium (Gibco) that contained 10% FBS (HyClone). Another RCC cell line, A498, was kindly gifted from Professor Jinhua Yang (Zhengzhou University) and also maintained in RPMI‐1640 medium. In addition, the RCC cell line SN12‐PM6 and human renal proximal tubular cell line HK‐2 were kind gifts from Dr Xiaoping Zhang (Union Hospital) and cultured in DMEM (Gibco) containing 10% FBS. These cells were placed at 37°C under humidified air containing 5% CO_2_.

### 2.3 Quantitative real‐time PCR (qRT‐PCR)

TRIzol reagent (Invitrogen) was utilized to isolate total RNA from ccRCC tissues and cell lines. For qRT‐PCR, 2 μg of DNase I‐treated RNA was used to synthesize cDNA using a PrimeScript RT‐polymerase kit (Takara). The qRT‐PCR assay was conducted on a StepOnePlus^TM^ Real‐Time PCR system (Applied Biosystems) using SYBR Green (Takara). The internal controls were GAPDH and U6. Specific primers for GAPDH, SNHG5, ZEB1, CDH11, SEMA4C, YAP1, CADM1, PTEN, and VEGFA were acquired from Sangon (Shanghai, China). For primer sequences see Table S1. Primers for U6, miR‐205‐5p and other candidate miRNAs were procured from RiboBio (Guangzhou). Relative RNA abundance was determined by using the 2^−ΔΔCT^ method.

RETRACTED

### 2.4 Cell transfection

Small interfering RNAs (siRNAs) for SNHG5 and ZEB1 and control siRNA were provided by RiboBio. The siRNA sequences were as below: si‐SNHG5, 5′‐AGUAAUAACAAAAAGGAACAU‐3′; si‐ZEB1, 5′‐GGATAAAGAGATGGAAGAA‐3′. miR‐205‐5p mimic, NC mimic, miR‐205‐5p inhibitor and NC inhibitor were also provided by RiboBio. A SNHG5 overexpression vector (pcDNA3.1/SNHG5) and empty vector (pcDNA3.1/Control) were obtained from GeneChem Co.. Vectors containing short hairpin RNAs targeting SNHG5 (sh‐SNHG5) and negative control vector (sh‐NC) were also provided by GeneChem Co.. The sequences of sh‐SNHG5 and SNHG5 overexpressing vectors are listed in Table S1. Lipofectamine 2000 (Invitrogen) was used to transfect the above RNA oligoribonucleotides or constructs into ccRCC cells following the manufacturer's recommendation.

### 2.5 Western blotting

RIPA buffer (Thermo Scientific) was utilized to isolate the proteins in ccRCC specimens and cell lines. To prevent protein degradation, RIPA buffer was prepared with protease inhibitor cocktail (Beyotime Institute of Biotechnology). The collected proteins were then quantified with a bicinchoninicacid (BCA) kit (Beyotime Institute of Biotechnology) and subjected to western blotting. Anti‐ZEB1 antibody (ab124512) was acquired from Abcam. The antibodies against E‐cadherin (#4065), vimentin (#3932), MMP2 (#4022), and GAPDH (D16H11) were procured from Cell Signaling Technology. Secondary antibodies were acquired from Wuhan Boster Bioengineering Co.. The protein levels of different genes were analyzed via Image J software version 1.36b (https://imagej.nih.gov/ij/).

### 2.6 Fluorescence in situ hybridization (FISH)

The subcellular location of SNHG5 in ccRCC cells was determined by FISH. Fluorescein‐labeled antisense RNA probes specific for SNHG5 were procured from GenePharma Co. A sense RNA probe specific for SNHG5 served as a negative control. These tests were then carried out with the provided instruction manual.

### 2.7 Cell Counting Kit‐8 (CCK‐8) assay

Cells were inoculated at a density of 1.0 × 10^3^ cells/well into a 96‐pore plate, and then cultivated for 24, 48, 72, or 96 hours. Cell viability was evaluated using a CCK‐8 kit (Dojindo, Japan) following the supplier's protocols. The absorbance at 450 nm was recorded using a spectrophotometer.

RETRACTED

### 2.8 Wound‐healing assay

The ccRCC cells at the appropriate confluence were plated onto six‐well plates. A pipette tip was utilized to create a wound on monolayer cells. After wounding, the extent of cell migration was calculated, and the plates were photographed at 24 hours. Representative micrographs from the wound‐healing assay in cancer cells were then acquired.

### 2.9 Migration and invasion assays

In a 24‐well plate Transwell system, 5 × 10^4^ ccRCC cells were cultivated in the top chambers with uncoated membrane (for migration) or Matrigel‐coated membrane (for invasion) (8‐μm pore size, BD Biosciences, USA). The capabilities of ccRCC cell migration and invasion were then investigated following the supplier's instructions. Migrated or invaded cells were fixed in PBS containing 4% paraformaldehyde and then incubated with crystal violet solution. A light microscope (Olympus) was employed to count the cells and take pictures.

### 2.10 Flat plate clone formation test

After transfection, ACHN and 786‐O cells were placed into six‐well dishes at a concentration of 300/well. Colony formation was detected as previously described.^17^ Groups of more than 10 cells were defined as colonies; these colonies were dyed with crystal violet (0.1%) and counted. Plating efficiency was defined as the total number of positive colonies/initial number of inoculated cells × 100%.

### 2.11 Luciferase reporter gene assay

Synthetic fragments of SNHG5 sequence with the predicted binding sites of miR‐205‐5p or mutant type and ZEB1 3′‐untranslated region (UTR) sequences with wild‐type or mutant miR‐205‐5p‐binding sites were cloned into pMIR‐REPORT luciferase plasmids. Then, the above vectors and synthetic oligonucleotides were cotransfected into ccRCC cells. After transfection for 24 hours, the cells were harvested and tested with a luciferase assay kit (Promega) following the supplier's recommendations.

### 2.12 RNA immunoprecipitation (RIP) assay

RIP assay was conducted by utilizing an EZ‐Magna RIP™ RNA‐Binding Protein Immunoprecipitation Kit (Millipore). In short, ccRCC cells were lysed with a RIP lysis buffer following the manufacturer's protocols. Then, magnetic beads preincubated with antibodies were used to immunoprecipitate RNAs from the cell lysate supernatant at 4°C for 6 hours. The purified RNAs were identified by qRT‐PCR.

### 2.13 Animal experiments

ACHN cells (4 × 10^6^) stably expressing sh‐SNHG5, sh‐NC, pcDNA3.1/SNHG5, or pcDNA3.1/Con were implanted subcutaneously in female nude mice (aged 5 weeks, n* = *5 in each group). The mice were killed after five weeks, and tumor weight and size were measured. Meanwhile, each nude mouse was injected with the indicated cell lines (2 × 10^6^) through tail vein. The mice were executed six weeks later, and their lungs were collected for further examination. All mice were kept and fed under specific pathogen‐free conditions that had been approved by the Animal Care and Use Committee of Tongji Medical College. Hematoxylin‐eosin (HE) staining was conducted using standard methods to detect metastatic nodules in rat lungs.

RETRACTED

### 2.14 Statistical analysis

Statistics were calculated utilizing GraphPad Prism 6. Data are displayed as means ± standard deviation (*SD*). Student's *t* test, analysis of variance, Spearman correlation test, and chi‐squared test were used when appropriate. *P* < .05 was regarded as significant.

## 3 RESULTS

### 3.1 SNHG5 expression is enhanced in ccRCC and is correlated with disease progression

To determine whether SNHG5 is differentially expressed in ccRCC tissues, RNA sequencing data from ccRCC and nontumor kidney tissues downloaded from TCGA were analyzed. As shown in Figure 1A, A set of lncRNAs were observed differentially expressed in ccRCC and nontumor kidney tissues. Among them, SNHG5 owing to its relatively high abundance, was chosen for further study. After analysis of microarray datasets from TCGA, SNHG5 expression was found to be remarkably increased in ccRCC samples (Figure 1B). The results of qRT‐PCR analysis of 52 paired ccRCC specimens and matched nontumor kidney specimens were consistent, and as described in Figure 1C, SNHG5 abundance was obviously enhanced in the ccRCC samples examined in our study. Higher expression levels of SNHG5 were also observed in the four ccRCC cell lines examined (ACHN, 786‐O, A498 and SN12‐PM6) as compared with HK‐2 cells (Figure 1D). FISH analysis further indicated that SNHG5 was more predominantly expressed in ccRCC cells than in HK‐2 cells. In addition, SNHG5 was preferentially distributed within the ccRCC cell cytoplasm. (Figure 1E). Moreover clinicopathological analysis revealed that a high abundance of SNHG5 was positively correlated with tumor‐node‐metastasis (TNM) stage, tumor size, lymphatic invasion, and distant metastasis, but was not correlated with other clinicopathological characteristics, including sex, age, and Fuhrman grade (Table 1). Together, these data may implicate the aberrant expression of SNHG5 in the tumorigenesis and progression of human ccRCC.

**Figure 1:** lncRNA SNHG5 is upregulated in human ccRCC. A, Heat map showing the hierarchical cluster of lncRNAs differentially transcribed in sixty‐eight paired ccRCC and nontumor kidney tissues from TCGA database. Red indicates upregulation; blue represents downregulation. The red box represents SNHG5. B, SNHG5 expression levels in ccRCC (n = 542) and nontumor (n = 68) tissues based on TCGA dataset were compared. C, Relative expression of SNHG5 in 52 paired ccRCC and nontumor kidney tissues. D, The abundance of SNHG5 in four ccRCC cell lines and HK‐2 cells. E, Representative pictures showing the localization of SNHG5 in ccRCC cells (ACHN and 786‐O) and HK‐2 cells (scale bar = 10 µm). Each experiment was repeated in triplicate. Data represent means ± *SD*. ^*^ *P* < .05, ^**^ *P* < .01

RETRACTED

### 3.2 SNHG5 is required for the proliferation, migration, and invasion of ccRCC cells

To evaluate the potential effect of SNHG5 on the biological activity of ccRCC cells, SNHG5 was silenced in ACHN cells because of their relatively high endogenous expression of SNHG5. Owing to the relatively low abundance of SNHG5 in 786‐O cells, SNHG5 expression was restored in 786‐O cells to explore the function of SNHG5. As presented in Figure 2A, SNHG5 expression was substantially reduced in the siRNA‐mediated knockdown group compared to the scrambled negative control (si‐Control) group of ACHN cells. In contrast, transfection of the pcDNA3.1/SNHG5 vector led to a higher expression of SNHG5 in 786‐O cells. The CCK‐8 assay revealed that SNHG5 silencing markedly repressed the proliferation of ACHN cells, whereas the ectopic overexpression of SNHG5 promoted the proliferative ability of 786‐O cells (Figure 2B,C). Subsequently, wound‐healing experiments indicated that the silencing of SNHG5 remarkably hampered the migration of ACHN cells, while SNHG5 overexpression enhanced the migratory abilities of 786‐O cells (Figure 2D). Consistent with the above data, the Transwell assay revealed that SNHG5 silencing robustly inhibited the migratory and invasive capabilities of ACHN cells compared to those of the control group, while overexpressed SNHG5 dramatically increased the migratory and invasive capacities of 786‐O cells (Figure 2E). The potential regulatory effect of SNHG5 on cell phenotype was also investigated in ccRCC cells. An EMT‐like phenotype was induced by SNHG5 silencing in ACHN cells, whereas SNHG5 overexpression exerted the opposite effect on 786‐O cells (Figure 2F). In the flat plate clone formation assay, knockdown of SNHG5 obviously inhibited the formation of ACHN cell colonies, whereas restoration of SNHG5 significantly facilitated the formation of 786‐O cell colonies (Figure 2G). We further assessed EMT‐related proteins in transfected cells. The data indicated that downregulation of SNHG5 led to an increased protein level of E‐cadherin but decreased protein levels of ZEB1, MMP2 and vimentin in ACHN cells. Conversely, restoration of SNHG5 had the opposite effect on 786‐O cells (Figure 2H). These outcomes suggest that SNHG5 can promote ccRCC progression by affecting cell proliferation, migration, and invasion.

RETRACTED

**Figure 2:** SNHG5 modulates the proliferation, migration, and invasion of ccRCC cells. A, The expression levels of SNHG5 in ACHN and 786‐O ccRCC cell lines transfected with si‐SNHG5 or pcDNA3.1/SNHG5 vector were analyzed using qRT‐PCR. B, C, CCK‐8 assay of ccRCC cells transfected with si‐SNHG5 or pcDNA3.1/SNHG5 vector. D, Representative wound closure images in SNHG5‐knockdown or SNHG5‐overexpressing ccRCC cell lines. Scale bar = 200 µm. E, Transwell experiments showed cell migration and invasion capability in ccRCC cell lines following transfection with si‐SNHG5 or pcDNA3.1/SNHG5 vector. Scale bar = 50 µm. F, Changes in EMT‐associated cell morphology in ccRCC cell lines transfected with si‐SNHG5 or pcDNA3.1/SNHG5 vector. Scale bar = 20 µm. G, Clonogenic assay in ccRCC cell lines transfected with si‐SNHG5 or pcDNA3.1/SNHG5 plasmids for 2 wks. H, Western blots for ZEB1, vimentin, E‐cadherin, and MMP2 in ccRCC cell lines following knockdown or overexpression of SNHG5. Data indicate means ± SD. ^*^ *P* < .05, ^**^ *P* < .01

### 3.3 SNHG5 regulates tumorigenicity and metastasis in vivo

To unravel whether SNHG5 is implicated in the tumorigenesis of ccRCC in vivo, ACHN cells with stable transfection of sh‐NC, sh‐SNHG5, pcDNA3.1/Con, or pcDNA3.1/SNHG5 vector were subcutaneously implanted into nude mice. SNHG5 silencing significantly suppressed tumor cell growth in vivo and exerted an obvious reduction in tumor volume and weight as compared with those of the control group (sh‐NC); however, the transfection of ccRCC cells with pcDNA3.1/SNHG5 vector had an opposite effect when compared with the control group (Figure 3A‐C). Meanwhile, a pulmonary metastasis model of ccRCC cells in nude mice was used to investigate the function of SNHG5. The number of pulmonary metastatic nodules was markedly reduced in the SNHG5‐knockdown group as compared with the control group. Additionally, overexpression of SNHG5 showed an obvious increase in pulmonary metastatic nodules compared to controls (Figure 3D,E). These findings revealed that SNHG5 regulates tumorigenicity and metastasis in ccRCC cells.

**Figure 3:** SNHG5 regulates ccRCC cell growth and lung metastasis in vivo. A, Photographs of representative tumor xenografts in nude mice that underwent subcutaneous implantation with sh‐NC‐, sh‐SNHG5‐, pcDNA3.1/Con‐, or pcDNA3.1/SNHG5‐transfected ACHN cells after 4 wks. Tumor volume B, and tumor weight C, were compared. D, Representative sections from pulmonary metastatic model mice and pathological pictures of metastatic nodules in the lung stained with HE. The blue arrows indicate tumor nodules. Upper layer: scale bar = 100 μm; lower layer: scale bar = 30 μm. E, Metastases in the lung were counted. Data represent means ± *SD*. ^*^ *P* < .05, ^**^ *P* < .01

RETRACTED

### 3.4 SNHG5 functions as a competing ceRNA for miR‐205‐5p

Evidence has shown that lncRNAs can function as ceRNAs and interact with miRNAs. To investigate whether SNHG5 possesses similar mechanism in ccRCC, we used StarBase^18^ and DIANA‐LncBase^19^ to predict the potential miRNAs regulated by SNHG5. Seventeen miRNAs were selected for further investigation. A qRT‐PCR assay was applied to validate the expression levels of candidate miRNAs in ccRCC cells transfected with si‐SNHG5, si‐NC, pcDNA3.1/SNHG5, or pcDNA3.1/Con. The results revealed that only miR‐205‐5p expression exhibited an obvious change in both transfected ccRCC cell lines (Figure 4A,B). As described in Figure 4C, a strong immunoprecipitation signal for the Ago2 protein was observed in extracts of ACHN cells. Simultaneously, the expression levels of SNHG5 and miR‐205‐5p in immunoprecipitates were examined using qRT‐PCR. Both SNHG5 and miR‐205‐5p were highly enriched in Ago2 immunoprecipitates compared to control IgG immunoprecipitates. Of note, low expression of miR‐205‐5p was observed in the four ccRCC‐derived cell lines examined (ACHN, 786‐O, A498, and SN12‐PM6) than in HK‐2 cells (Figure 4D). Moreover StarBase, DIANA, PicTar and TargetScan Human 7.1 were taken to predict potential targets modulated by miR‐205‐5p. Seven candidate target genes (CDH11, SEMA4C, YAP1, CADM1, PTEN, ZEB1, and VEGFA) were selected for further investigation. Interestingly, ZEB1 transcript was the only one among the analyzed candidates that were differentially expressed in miR‐205‐5p mimic‐transfected ACHN cells or miR‐205‐5p inhibitor‐transfected 786‐O cells (Figure 4E,F). Furthermore, the expression of ZEB1 mRNA in ACHN cells was found to be obviously downregulated after knockdown of SNHG5 by siRNA, whereas the expression of ZEB1 mRNA in 786‐O cells was remarkably upregulated by ectopic overexpression of SNHG5 (Figure 4G). Additionally, the restoration of miR‐205‐5p markedly reduced ZEB1 protein expression in ACHN cells. In contrast, the knockdown of miR‐205‐5p significantly increased the protein expression of ZEB1 in 786‐O cells (Figure 4H). To determine the functional associations among SNHG5, miR‐205‐5p, and ZEB1 in ccRCC cells, we conducted a luciferase assay. As shown in Figure 4I, SNHG5 harbors potential binding sites for miR‐205‐5p, which contains potential binding sites within the 3′‐UTR of ZEB1. Compared to luciferase reporter activity in the control group, luciferase activity was markedly inhibited in ACHN cells cotransfected with SNHG5‐wt plasmid and miR‐205‐5p mimic. After the cotransfection of miR‐205‐5p inhibitor and SNHG5‐wt plasmid into ACHN cells, luciferase activity in wild type group was dramatically enhanced compared to the control group. Nevertheless, these effects were robustly reversed after mutating the putative binding sites of miR‐205‐5p (Figure 4J). Similarly, luciferase activity of ccRCC cells cotransfected with wild‐type ZEB1 3′‐UTR reporter vector (ZEB1‐wt) and miR‐205‐5p mimic was markedly impaired, but cotransfection with miR‐205‐5p inhibitor obviously increased luciferase activity in ccRCC cells. However, transfection with reporter vector harboring a mutant ZEB1 3′‐UTR sequence (ZEB1‐mut) in which putative miR‐205‐5p‐targeted sites had been mutated abrogated the above effects (Figure 4K). Else, we checked miR‐205‐5p expression in matched ccRCC and nontumor kidney tissues. The data revealed that a lower miR‐205‐5p expression was observed in ccRCC tissues than in nontumor kidney tissues (Figure 4L). Further analysis showed a negative Pearson's correlation between the expressions of miR‐205‐5p and SNHG5 in ccRCC tissues (Figure 4M). Moreover ZEB1 mRNA was obviously increased in ccRCC tissues compared to nontumor kidney tissues (Figure 4N). Pearson's correlation analyses showed that the level of ZEB1 mRNA was inversely correlated with miR‐205‐5p expression and positively correlated with SNHG5 expression in ccRCC tissues (Figure 4O,P). Altogether, the results showed that SNHG5 may serve as a ceRNA to sponge miR‐205‐5p and thus regulates ZEB1 expression.

RETRACTED

**Figure 4:** SNHG5 functions as a ceRNA to regulate ZEB1 expression via competitively binding miR‐205‐5p. A, B, qRT‐PCR was employed to examine the expression levels of candidate miRNAs in two ccRCC cell lines (ACHN and 786‐O) following transfection with si‐SNHG5 or pcDNA3.1/SNHG5 vector. C, RNA immunoprecipitation (RIP) analysis validated the close correlation between miR‐205‐5p and SNHG5 in ACHN cells. D, miR‐205‐5p expression level in different ccRCC cell lines was detected using qRT‐PCR. U6 was used as a control. E, F, qRT‐PCR was applied to check the mRNA levels of predicted miR‐205‐5p targets in ccRCC cell lines following transfection with miR‐205‐5p mimic or miR‐205‐5p inhibitor. G, qRT‐PCR analysis showing ZEB1 mRNA levels in si‐SNHG5‐transfected ACHN cells and pcDNA3.1/SNHG5‐transfected 786‐O cells. H, Western blotting was performed to check ZEB1 protein level in ccRCC cell lines after overexpression or knockdown of miR‐205‐5p. I, Putative miR‐205‐5p‐binding sites in wild type/mutant SNHG5 or ZEB1 3′‐UTR sequences. J, K, Analysis of luciferase activity to determine the potential association among SNHG5, miR‐205‐5p and the ZEB1 3′‐UTR. L, qRT‐PCR examination of miR‐205‐5p expression in 52 pairs of ccRCC tissues and normal kidney tissues. M, Negative association between SNHG5 and miR‐205‐5p level in ccRCC tissues (n = 52). N, qRT‐PCR was performed to analyze the mRNA expression of ZEB1 in 52 ccRCC tissues and matched normal kidney tissues. O, Negative correlation between ZEB1 and miR‐205‐5p expression in ccRCC tissues (n = 52). P, Positive correlation between SNHG5 and ZEB1 expression in ccRCC tissues (n = 52). Data are means ± SD. ^*^ *P* < .05, ^**^ *P* < .01

### 3.5 SNHG5 enhances ccRCC cell proliferation, migration, and invasion by inhibiting the miR‐205‐5p/ZEB1 axis

To investigate whether SNHG5 exerts its effects in ccRCC cells via miR‐205‐5p, a rescue assay was performed. SNHG5 inhibition obviously repressed the proliferation, migration, invasion and colony formation of ACHN cells; nevertheless, these inhibitory effects could be attenuated by cotransfection with miR‐205‐5p inhibitors (Figure 5A‐G). In contrast, the ectopic overexpression of SNHG5 by pcDNA3.1/SNHG5 remarkably enhanced the capabilities of proliferation, migration, invasion, and colony formation of 786‐O cells. Restoration of miR‐205‐5p by transfection with miR‐205‐5p mimic reversed the effects induced by SNHG5 overexpression (Figure 5A‐G). Notably, we further confirmed the tumor‐suppressive effect of miR‐205‐5p in ccRCC cells. Moreover, western blot analysis of the EMT‐related marker ZEB1 indicated that the reduced protein level of ZEB1, induced by SNHG5 knockdown, was restored by the cotransfection with miR‐205‐5p inhibitor in ACHN cells (Figure 5H,I). In contrast, SNHG5 overexpression enhanced the expression of ZEB1; nevertheless, this enhanced expression was attenuated by cotransfection with miR‐205‐5p mimic in 786‐O cells (Figure 5H,I). These data revealed that SNHG5 facilitated the malignant behaviors of ccRCC cells in a miR‐205‐5p‐dependent manner. We then investigated the regulation of ccRCC proliferation, migration, invasion and colony formation by SNHG5 and ZEB1. Restoration of SNHG5 enhanced the proliferation and colony formation of ccRCC cells and facilitated ccRCC cell migration and invasion; however, these promotive effects were attenuated by ZEB1 knockdown (Figure 6A‐F). Consistent with the above results, the increased expression of ZEB1 in ccRCC cells, induced by the restoration of SNHG5, could also be reversed by cotransfection with si‐ZEB1 (Figure 6G,H). Altogether, the above data suggested that SNHG5 regulates ccRCC cell proliferation, migration, and invasion via the miR‐205‐5p/ZEB1 axis.

RETRACTED

**Figure 5:** SNHG5 modulates ccRCC cell proliferation, migration, and invasion in a miR‐205‐5p‐dependent manner. A, CCK‐8 assay of the proliferative activities in ACHN and 786‐O cell lines cotransfected with si‐con and miR‐205‐5p inhibitor, si‐SNHG5 and miR‐205‐5p inhibitor, pcDNA3.1/con and miR‐205‐5p mimic, or pcDNA3.1/SNHG5 and miR‐205‐5p mimic. B‐E, Transwell assays showed that SNHG5 expression restored the suppressive effect of miR‐205‐5p on the migratory and invasive capacities of ccRCC cell lines. Scale bar = 50 µm. F, G, Clonogenic assay in ccRCC cell lines after cotransfection. H, I, Western blot analysis of ZEB1 protein in cotransfected ccRCC cell lines. Data show means ± SD. ^*^ *P* < .05, ^**^ *P* < .01

**Figure 6:** SNHG5 facilitates ccRCC cell proliferation, migration, and invasion via ZEB1. A, CCK‐8 assay of the proliferative activities of 786‐O cells following cotransfection with si‐ZEB1 and pcDNA3.1/con or si‐ZEB1 and pcDNA3.1/SNHG5. B‐D, Transwell assays demonstrated that the effect of pcDNA3.1/SNHG5 in promoting migration and invasion was reversed by ZEB1 silencing in 786‐O cells. Scale bar = 50 µm. E, F, Colony formation assay of 786‐O cells following cotransfection with si‐ZEB1 and pcDNA3.1/con or si‐ZEB1 and pcDNA3.1/SNHG5. G, H, Western blots for ZEB1 in 786‐O cells after cotransfection. Data reflect means ± SD. ^*^ *P* < .05, ^**^ *P* < .01

## 4 DISCUSSION

In recent decades, increasing evidence has uncovered the key roles of lncRNAs in various human malignances, including ccRCC.^5^, ^20^, ^21^ These findings are of benefit to elucidate the mechanistic basis of ccRCC; nevertheless, only a small proportion of lncRNAs and their functions have been revealed. The identification of novel lncRNAs and exploration of the underlying mechanism of ccRCC progression still require a substantial amount of research. LncRNA SNHG5 resides in the introns of host genes and was recently identified to play a vital role in several kinds of human malignances. In bladder cancer, SNHG5 was demonstrated to promote the cellular proliferation of cancer cells and high expression of SNHG5 was closely correlated to poor prognosis.^13^ SNHG5 expression was identified to be elevated in colorectal cancer, and overexpression of SNHG5 was verified to facilitate cancer cell survival and migration.^14^ Conversely, SNHG5 was shown to suppress gastric cancer (GC) cell proliferation and metastasis via interaction with MTA2.^22^ The contradictory functions of SNHG5 in different types of cancers may be attributed to the tissue‐specific expression and functional structures of lncRNAs. In this study, we showed that the expression level of SNHG5 was markedly elevated in ccRCC tissues and different ccRCC cell lines. Specifically, several clinicopathological features of ccRCC patients (tumor size, TNM stage, lymph node invasion and distant organ metastasis) were closely associated with high SNHG5 expression levels, potentially implicating SNHG5 in the pathogenesis and progression of ccRCC. We further found that SNHG5 promoted ccRCC cell proliferation, migration, invasion, EMT, and growth*.* These experiments revealed that SNHG5 harbors an oncogenic function in the modulation of the properties of ccRCC.

RETRACTED

Although we have confirmed the oncogenic function of SNHG5 in ccRCC, the detailed molecular mechanism by which SNHG5 is involved in carcinogenesis and progression requires further exploration. In recent years, increasing evidence has implicated lncRNAs in a network of interacting ceRNAs, which bind miRNAs and inhibit miRNAs binding to their target genes in human cancers.^23^ For instance, the lncRNA PCAT6 was identified as a ceRNA for miR‐204 that thereby enhances colorectal cancer cell chemoresistance through modulating HMGA2.^24^ Another mechanistic investigation confirmed that the lncRNA H19 acts as a miR‐141 sponge to activate the β‐catenin pathway which is involved in colorectal cancer chemoresistance.^25^ Additionally, the lncRNA ARNILA was demonstrated to facilitate breast cancer invasion and metastasis through the ARNILA/miR‐204/Sox4 signaling pathway.^26^ Strikingly, as a miR‐26a‐5p sponge, SNHG5 was confirmed to upregulate the expression of GSK3β in hepatocellular carcinoma.^15^ Moreover, the SNHG5/miR‐32/KLF4 axis was shown to be implicated in the modulation of cell proliferation and migration in gastric cancer.^27^ Thus, in our study, we sought to determine whether SNHG5 may also serve as a ceRNA to modulate the tumorigenesis and progression of ccRCC. Using bioinformatics database (starBase^18^ and DIANA LncBase^19^), we found that SNHG5 contained potential miR‐205‐5p binding sites. As expected, SNHG5 was demonstrated to directly bind to miR‐205‐5p and attenuate the expression level of miR‐205‐5p in ccRCC cells. Recent reports have shown the tumor suppressive effect of miR‐205‐5p in several human tumors.^11^, ^28^, ^29^ Consistent with previous findings, the downregulated expression of miR‐205‐5p in ccRCC specimens and cell lines and the tumor‐suppressive function of miR‐205‐5p were further confirmed in our study. Additionally, Pearson correlation analysis revealed that miR‐205‐5p was inversely associated with the abundance of SNHG5 in ccRCC samples. Importantly, SNHG5 and miR‐205‐5p in the Ago2‐containing RNA‐induced silencing complex (RISC) were also shown to be positively correlated by RIP analysis. Based on these findings, we concluded that SNHG5 can competitively interact with miR‐205‐5p and inhibit the expression of miR‐205‐5p in ccRCC. Moreover the biological function of SNHG5 in ccRCC cells is mediated by miR‐205‐5p, as shown by our rescue experiment. These results are consistent with our hypothesis and previous report^16^ indicating that SNHG5 binds miR‐205‐5p and affects the expression and function of miR‐205‐5p in ccRCC.

RETRACTED

We further investigated the downstream target of miR‐205‐5p and function of SNHG5 on the biological activity of ccRCC. Among various invasion‐ and metastasis‐related mechanisms, EMT has been well studied in different kinds of human cancers, including ccRCC.^30^ According to current knowledge, EMT is an essential step that facilitates the transition of tumor cells to a mesenchymal phenotype and facilitates tumor cells invasion and metastasis.^31^ ZEB1, an EMT‐inducing zinc finger transcription factor, is overexpressed in various cancers and promotes EMT and tumor initiation, growth, invasion and metastasis.^32^ Notably, recent reports have shown that lncRNAs are implicated in modulation of the miRNA/ZEB1 axis in human carcinomas. For example, the lncRNA ZFAS1 was found to counteract miR‐150 and activate ZEB1 expression in hepatocellular carcinoma.^33^ The lncRNA PTAR was shown to be involved in EMT and the malignant transformation of serous ovarian cancer cells via interaction with the miR‐101‐3p/ZEB1 axis.^34^ Here, the present data showed that SNHG5 could increase the expression of ZEB1 by sequestering endogenous miR‐205‐5p in ccRCC cell lines. Simultaneous correlation analysis indicated that ZEB1 mRNA level was inversely correlated with miR‐205‐5p but positively correlated with SNHG5 in ccRCC tissues. ZEB1 was eventually verified to be a direct target of miR‐205‐5p in ccRCC. Together, these outcomes indicated that SNHG5 serves as a ceRNA that binds miR‐205‐5p and abrogates miR‐205‐5p‐induced inhibition of ZEB1 in ccRCC. Furthermore, rescue experiments revealed that SNHG5 modulates the malignant biological behaviors of ccRCC cells via the miR‐205‐5p/ZEB1 axis. We therefore present a model that SNHG5 promotes the progression of EMT and tumor proliferation, migration, invasion and metastasis cascade by elevating ZEB1 expression through binding miR‐205‐5p in ccRCC (Figure 7).

**Figure 7:** A proposed schematic ceRNA model to summarize the SNHG5/miR‐205‐5p/ZEB1 pathway. SNHG5 can increase the expression level of ZEB1 via competitively binding miR‐205‐5p. Subsequently, ZEB1 upregulation facilitates ccRCC growth and induces EMT, eventually promoting the migration, invasion, and metastasis of ccRCC cells

To conclude, this study provides promising evidence that high SNHG5 expression contributes to ccRCC progression. miR‐205‐5p was demonstrated to act as not only a direct target of SNHG5 but also a mediator of SNHG5 in ccRCC cells. miR‐205‐5p was further identified to target ZEB1, which modulated the biological functions of ccRCC cells by promoting proliferation and inducing tumor EMT. A SNHG5/miR‐205‐5p/ZEB1 signaling axis was presented to uncover the underlying mechanism of tumorigenesis and progression in ccRCC; this axis also offers potential therapeutic targets against ccRCC.

RETRACTED

## CONFLICT OF INTEREST

None.

## AUTHOR CONTRIBUTIONS

Chuanhua Zhang conceptualized and designed the study. Lei Lv collected the tissue samples and acquired the data. Wei Xiang and Gaofeng Zhou performed the in vitro and in vivo assays.Wei Wu analyzed the statistical data. Jingdong Yuan provided technical or material support. Chuanhua Zhang and Guosong Jiang revised and approvedthe final manuscript.

## Supporting information

Table S1

## Data Availability

All data used to support the findings of this study are available upon request by contact with the corresponding author.
